# Knockdown of Long Noncoding RNA LINC00240 Inhibits Esophageal Cancer Progression by Regulating miR-26a-5p

**DOI:** 10.1155/2022/1071627

**Published:** 2022-10-05

**Authors:** Yupeng Liu, Tao Li, Chunlei Peng, Qinghua Mao, Biao Shen, Minxin Shi, Haimin Lu, Ting Xiao, Aimin Yang, Chun Cheng

**Affiliations:** ^1^Department of Thoracic Surgery, Tumor Hospital Affiliated to Nantong University, Nantong 226000, China; ^2^Department of Medical Oncology, Tumor Hospital Affiliated to Nantong University, Nantong 226000, China

## Abstract

**Background:**

Esophageal cancer is the most prevalent digestive system tumor. Due to a lack of characteristic symptoms and early diagnosis, a confirmed esophageal cancer is typically detected at a progressively harmful stage. Therefore, it is critical to investigate the molecular mechanisms governing the formation and progression of esophageal cancer in order to identify new treatment targets for esophageal cancer early detection.

**Methods:**

We first screened the differentially expressed gene LINC00240 in the TCGA database. Multivariate analysis and Cox regression were performed, and a nomogram was constructed for internal validation. The correlation between LINC00240 and immune cells was analyzed using the TIMER database. The possible mechanism of action was explored through GSEA enrichment analysis. Then, in 43 esophageal cancer tissues, paracancour tissues, and cell lines, the LINC00240 expression was found. Transwell assays, CCK-8, and clone formation assays were utilized to assess the impact of LINC00240 on the metastasis of esophageal cancer cells. The binding activity of LINC00240 to downstream miRNAs was assessed using the luciferase reporter gene.

**Results:**

TCGA database showed that LINC00240 expression was increased in cancer tissues compared to adjacent tissues. The *C*-index of the nomogram is 0.712 (0.666–0.758), and the prediction model has good accuracy. According to the TIMER database, the LINC00240 expression is linked to immune infiltration and may be crucial in encouraging the immune escape of tumor cells. Gene enrichment analysis depicts that LINC00240 could influence the biological events of esophageal cancer by taking part in pathways such as affecting the cell cycle. LINC00240 expression was substantially greater in the plasma of esophageal cancer patients (3.94 ± 1.55) than in the normal control group (2.13 ± 0.89). Plasma expression of LINC00240 was linked to the degree of differentiation (*P*=0.0345) and TNM stage (*P*=0.0409). Knocked down LINC00240 inhibited esophageal cancer cells proliferation, lone formation, and invasion. LINC00240 might bind itself to miR-26a-5p and influence its expression. MiR-26a-5p inhibitor can dramatically limit the ability of LINC00240 knockdown on plate colony formation and relocation of esophageal cancerous cells was demonstrated in colony formation and migration experiments.

**Conclusion:**

LINC00240 expression is elevated in esophageal cancerous tissues, and knocking down LINC00240 decreases esophageal cancer cell proliferation, clone formation, invasion, and migration via miR-26a-5p. As a result, LINC00240 could be a novel target for esophageal cancer patients' early diagnosis and treatment.

## 1. Introduction

Esophageal cancer (EC) is the world's sixth greatest reason behind deaths related to cancer and the eighth most common type of cancer. Esophageal squamous cell carcinoma (ESCC) and esophageal adenocarcinoma (EA) are among the two most common forms of EC [1]. Considering the advancements in the pharmacological therapies for treating EC, tens of thousands of people still die from esophageal cancer every year worldwide, and the incidence of esophageal cancer remains high in China [2, 3]. The main treatment method is surgery along with radiation and chemotherapy for esophageal cancer at present, yet the limitations of surgical treatment and many adverse reactions of radiotherapy and chemotherapy combined with the fact that most patients are diagnosed in an advance stage result in a low survival rate and physical and mental burden of patients [4, 5]. Therefore, finding new early diagnostic biomarkers or therapeutic targets is one of the main goals of EC research to prolong the survival of patients.

lncRNAs (long noncoding RNAs) are a form of RNA with over 200 nucleotides and occupy at least 80% of the human genome but do not code for proteins [6]. According to growing data, many biological functions, including proliferation, metastasis, cell cycle progression, cell development, and apoptosis, are thought to be influenced by lncRNAs [7, 8]. In the process of gene modification, lncRNAs act as transcriptional regulators, posttranscriptional processing factors, chromatin remodelers, and splicing regulators [9]. In addition, lncRNAs take part in the detection and therapy of cancers and in promoting or inhibiting cancer development. The use of lncRNA as a ceRNA to control the progression of esophageal cancer has been a hot topic in the study, and it could be a possible oncogene or tumor suppressor gene involved in the biological process of the disease; for example, lncRNA DNM3OS secreted by cancer-associated fibroblasts increases radioresistance by modulating DNA destruction in ESCC [10]. lncRNA EIF3J-AS1 increases AKT1 mRNA levels through miR-373-3p, thus exhibiting oncogenic function in EC, and can serve as a possible treatment target and prognostic biomarker [11]. Therefore, in-depth exploration of the functions or regulatory pathways of lncRNAs in esophageal cancer will provide a theoretical basis and possible targets for timely detection and treatment of esophageal cancer.

LINC00240 is a new class of lncRNAs identified in recent years and is responsible for manifesting various tumors, such as gastric, liver, and cervical cancer [12–14]. But the function and LINC00240 molecular mechanism in tumor tissue, especially in esophageal cancer tissue, are still unclear. Our study mainly researched the expression of LINC00240 and its function in the biological events of esophageal cancer patients. In addition, bioinformatics analysis and *in vitro* experiments were performed to study the effects of LINC00240 on tumor cell behavior and its underlying mechanisms.

## 2. Material and Method

### 2.1. Data Analysis Using TCGA Database

The TCGA database was employed for data analysis to investigate the LINC00240 expression in esophageal cancer.

### 2.2. Construction and Evaluation of the Nomogram

To personalize the predicted survival probabilities at 1, 3, and 5 years, nomograms were constructed as per the outcomes of the multivariate analysis. The RMS *R* package was employed to construct nomograms. The discriminative power of the nomogram was assessed by employing the Concordance Index (*C*-index), which was calculated using the bootstrapping technique with 1000 resampling. Additionally, the *C*-index was utilized to compare the predictive accuracy of nomograms and specific prognostic factors.

### 2.3. Correlation between LINC00240 and Immune Cells in the TIMER Database

The correlation between the LINC00240 expression and various immune cells in esophageal cancer was illustrated by constructing a bar graph from the TIMER database.

### 2.4. GSEA Enrichment Analysis

Functional analysis was performed online using Metascape. Add differential genes to Metascape for functional analysis.

### 2.5. Clinical Sample Collection

Nantong Tumor Hospital's ethics committee accepted this study, and all participants signed informed consent forms (NO. 2022-A 05). A total of 43 preoperative plasma samples from patients with esophageal cancer in our hospital from January 2019 to June 2021 were collected, and 43 healthy control group plasma samples were also collected. In addition, a total of 43 pairs of postoperative tumor tissue and paracancours normal tissue samples were collected. Patients were in the 32 to 72 years old age range, with an average of 52.5 ± 8.12 years, and included 24 males and 19 females. All patients' tissue samples were pathologically diagnosed as esophageal cancer, with no antitumor treatment such as radiotherapy or chemotherapy before surgery. The paracancerous tissue is the normal tissue located 5 cm from the tumor tissue. The tissue obtained by surgical resection is washed with normal saline and immediately placed in liquid nitrogen for preservation. After adding RNA buffer, it was frozen via liquid nitrogen for later use, and total RNA in tissues was then extracted.

### 2.6. Cell Culture

Esophageal cancer (EC) cell lines (OE-33, KYSE-150, TE-10, and Eca-109) and human normal esophageal epithelial cells (HEEC) and KYSE-30 were bought from Shanghai Cell Center, Chinese Academy of Sciences, and experimentally preserved. All (EC) cells were grown in RPMI 1640 media (ScienCell, Carlsbad, CA, USA) with 10% fetal bovine serum (FBS) (Gibco, Carlsbad, CA, USA) and 100 units/mL of penicillin and 100 milligrams of streptomycin. The cells were cultivated in a 5% CO_2_ incubator at 37°C, with the media being replaced every two days.

### 2.7. Real-Time PCR

Trizol technique was utilized to isolate total RNA (Invitrogen, USA), and total RNA purity was determined using the Nanodrop 2000 and identified by nucleic acid electrophoresis. To avoid RNase contamination, all instruments were treated with de-RNase before the experiment, and the mortar was precooled with liquid nitrogen. The primers of LINC00240 and internal reference GAPDH are referenced in [14] and from GenePharma (Shanghai, China). The reaction was carried out by utilizing fluorescence quantitative PCR equipment with the reaction conditions listed below: predenaturation at 95°C for 15 seconds, followed by 45 cycles of denaturation at 95.0°C for 5 seconds, annealing, and extension at 60.0°C for 30 seconds. qRT-PCR was carried out with Bio-Rad iQ5 Real-Time PCR System SYBR Green kit (TaKaRa, Tokyo, Japan). The 2^−ΔΔCt^ method was employed for analyzing the expression difference between tumor tissue and paracancours normal tissue, where Ct was the number of amplification cycles required for the fluorescence intensity to reach the threshold, and the corresponding Ct value was calculated, ^Δ^Ct = Ct_LINC00240_ − Ct_GAPDH_, ^ΔΔ^Ct = ^Δ^Ct (normal tissue) − Ct (tumor tissue), and then the differences in the relative mRNA expression of each group were obtained.

### 2.8. Cell Transfection

In this study, the interfering sequence targeting LINC00240 was used as a reference [14]. The sequence was synthesized by Shanghai Sangong (Shanghai, China) and constructed into a lentiviral vector for subsequent transfection. Cells were digested with trypsin, 10 MOI of the virus was added to the medium, 400 *μ*l of serum-free medium Opti-MEM (Invitrogen, USA) was added in all the wells, and 100 microliters of the transfection solution prepared above was added, then the cells were incubated in 5% CO_2_ solution at 37°C and cultured in a carbon dioxide incubator. After culturing for 4–6 hours, carefully aspirate the culture medium with a pipette, and replace it with a new medium before continuing the culture.

### 2.9. Cell Viability Measurement by CCK8 Assay

After the transfection of esophageal cancer cells to all the groups, cells were counted after being cultured for 48 hours. The 96-well plates were transfected with cells at the density of 5 × 10^3^ cells per well. Every group had three duplicate wells, and only RPIM1640 was added to the zero-adjusted well. The medium was gently shaken and mixed and then cultured at 37°C in a 5% CO_2_ incubator. The CCK-8 (Beyotime, Beijing, China) was utilized to determine the cell viability at 0 d, 1 d, 2 d, and 3 d after culture. The detection process was executed completely as per the kit's accompanying manual: 10 *μ*l of CCK8 detection reagent was poured into all the wells along the well walls, and cells were incubated for 2 hours in a CO_2_ incubator. The OD value of all the wells was measured at 450 nm utilizing a microplate reader. The maximum and minimum values were removed, and the average of measurement results was utilized to build the growth curve.

### 2.10. Clone Formation Assay

After the transfection of esophageal cancer cells to all the groups, cells were counted after being cultured for 48 hours. About 800 cells in each group were transferred to a Petri dish and cultured in a carbon dioxide incubator. Every 2–3 days, the cell progression was monitored after changing the media. After culturing for about 14 days, the culture dish was taken out and twice washed in PBS buffer, and cells were fixed by adding 4% paraformaldehyde (Beyotime, Beijing, China) for 0.5 hours. The formaldehyde was removed by suction and washed twice with PBS buffer, and 4 ml of crystal violet staining solution (Beyotime, Beijing, China) was added for staining overnight at room temperature. Wash with PBS buffer 3–5 times after staining, and then collect photos of the formation of spots after drying. The number of clones is the cell mass of ≥50 cells, and the experiment is carried out three times.

### 2.11. Transwell Migration and Invasion Assay

Cell migration assay: take the cells in a good growth state, digest them with trypsin, and adjust the density to 1 × 106 cells/ml after cell counting. 500 *μ*l of culture media (having 20% FBS) was added to the Transwell chamber (8 *μ*m pore sizes, Corning, New York, USA), and 100 *μ*l of the cell suspension was injected into the upper Transwell chamber in a carbon dioxide constant temperature incubator for cultivation. Observation after culturing for 36 hours, aspirate the liquid that remains in the upper chamber, wash with PBS buffer three times, and clean the cells that have not been transferred in the upper chamber; add 600 *μ*l methanol to the cells transferred to the lower chamber for 30 minutes, and add 1% Crystal violet solution (Beyotime, Beijing, China) for staining. The cells were washed thrice in PBS buffer after staining, and five visual fields were picked at random for inspection under a light microscope, with the number of cells counted and statistically evaluated.

Cell invasion assay: dilute Matrigel gel (BD Biosciences, Bedford, MA) with serum-free medium RPIM-1640 at a 1 : 8 ratio, and cover the diluted gel into the inner base of the Transwell's upper chamber. Cells in a good growth state were taken, and the cell density was adjusted to 1 × 10^6^ cells/ml after cell counting. Add 500 *μ*l of medium (having 20% FBS) to the Transwell chamber, and inoculate 100 *μ*l of the cell suspension into the upper chamber. Avoid the formation of air bubbles during the procedure and make sure the cells are dispersed equally. Incubate in a carbon dioxide incubator at a steady temperature. After 36 hours of culture, observations are made, and data is processed and analyzed according to the migration experimental technique.

### 2.12. Dual-Luciferase Gene Activity Assay

To observe if the miR-26a-5p has targeted binding to the LINC00240 gene, we combined the luciferase reporter gene with 3′UTR of the wild-type LINC00240 and mutant LINC00240 genes and then combined miR-26a-5p with the 3′UTR of LINC00240 gene. Plasmids carrying the LINC00240 target segment were cotransfected into cells and cultured overnight in a carbon dioxide incubator. The Dual-Luciferase Reporter Assay System was employed to assess luciferase activity in cotransfected cells. The specific detection steps are as follows: discard the old cells in each well. The medium was washed three times with PBS buffer, 100 *μ*l of PLB (Passive Lysis Buffer) was added, and the cell lysate was collected after gently shaking to mix. Then 20 *μ*l lysate was added to the luminescent plate and detected with a GloMax bioluminescence detector. The measurement interval was set to 2 s and the measurement time was set to 10 s. Then 100 *μ*l of LAR I was added, the value was read for 2 s after rapid mixing, and the activity of hLuc luciferase was measured. The reporter gene cell lysate was used as a blank control group. Add 100 *μ*l Stop &Glo® Reagent (Promega, USA), mix quickly, and read for 2 s to measure hRluc luciferase activity. Taking hLuc/hRluc luciferase activity as the relative activity, the activation degree of the target reporter gene was compared according to the obtained ratio.

### 2.13. Statistical Analysis

SPSS 19.0 was employed to analyze the data; measurement data was represented as (mean ± standard deviation, ±*s*), and measurement data with a normal distribution were compared across groups using the *t*-test or (ANOVA) and nonparametric rank sum test. The chi-square test was employed to examine the enumeration data. A significant difference was set as *P* < 0.05.

## 3. Results

### 3.1. Elevated Expression of LINC00240 in Esophageal Cancer

We first performed a pan-cancer analysis through the TCGA database and observed that LINC00240 expression was elevated in most tumor tissues (Figure 1(a)). Further analysis revealed that LINC00240 expression was also elevated in esophageal cancer tumor tissues (Figure 1(b)). Constructing the ROC curve found that the AUC was 0.713, so LINC00240 also had a good prediction effect (Figure 1(c)).

### 3.2. Nomogram Construction

For individually predicting the 1, 3, and 5-year survival probability of esophageal cancer patients, we constructed a nomogram based on the outcomes of multivariate analysis in the TCGA database. The nomogram *C*-index was 0.712 (0.666–0.758), which predicted the model has good prediction accuracy (Figure 2).

### 3.3. Correlation among LINC00240 and Immune Cells in the TIMER Database

A bar graph was constructed showing the correlation between the LINC00240 expression and various immune cells in esophageal cancer using the TIMER database.

A significant link between the LINC00240 expression and most of the infiltrating immune cells was observed, including a positive correlation with NK cells, Tcm, Th2 cells, NK CD56dim cells, etc. It was also observed that Mast cells, DC cells, *B* cells, and neutrophils were negatively correlated (Figure 3(a)).

To further evaluate the influence of LINC00240 on the tumor microenvironment (TME), the correlation between the LINC00240 and specific immune cells was analyzed, and the outcomes revealed that different LINC00240 expressions correlated with the level of immune cell infiltration in most tumors (Figure 3(b)). These findings further support that LINC00240 expression could be considerably associated with immune infiltration and indicate that LINC00240 might have a significant function in promoting immune escape of tumor cells in the esophageal cancer tumor microenvironment, which also serves as a stronger resource for basic research in the future.

### 3.4. Correlation between LINC00240 and Drug Target Molecules in Molecular Targeted Therapy in TCGA Database

Considering the diversity of current treatments for esophageal cancer and the selectivity of current targeted therapy drugs, the NCCN guidelines also point out that targeted therapy drugs for esophageal cancer include anti-EGFR monoclonal antibodies such as nimotuzumab, or, for EGFR gene mutations, such as gefitinib and erlotinib. Targeted drugs also include specific antibodies against PD-1, such as so-called immune checkpoint inhibitors such as camrelizumab or toripalizumab. Targeted drugs also include targeted drugs against tumor angiogenesis, such as bevacizumab or recombinant human endostatin injection, that is, Endostat and so on. We conducted a correlation study between LINC00240 and the target molecules of these targeted drugs, and we found that LINC00240 had a good correlation with EGFR, VEGFA, VEGFB, VEGFC, VEGFD, ERBB2, and MSI1 (Figure 4).

### 3.5. Coexpression Gene Analysis of LINC00240

Data mining from the TCGA database was employed for identifying the positively or negatively correlated genes coexpressed with LINC00240. The graph illustrates the top 50 genes that are positively and negatively associated with LINC00240 in esophageal cancer (Figures 5(a) and 5(b)).

### 3.6. Prediction of GSEA-Based Signaling Pathways

We performed functional analysis online using Metascape. It was observed that LINC00240 might influence the biological events of esophageal cancer through these five pathways: KEGG_APOPTOSIS; KEGG_VEGF_SIGNALING_PATHWAY; WP_EGFEGFR_SIGNALING_PATHWAY; REACTOME_CELL_CYCLE_CHECKPOINTS; REACTOME_G2_M_DNA_DAMAGE_CHECKPOINT. The results of these predictions also provide a reference for the basic experimental research we carry out below (Figure 6).

### 3.7. LINC00240 Is Highly Expressed in Esophageal Cancer Tissues and Cell Lines

Fluorescence quantitative PCR was employed to determine LINC00240 expression in 43 esophageal cancer and paracancours tissues. In comparison to paracancours tissues, LINC00240 was shown to be strongly expressed in esophageal cancer tissues (Figure 7(a)). LINC00240 expression was detected by fluorescent quantitative PCR in esophageal cancer cell lines (OE-33, KYSE-150, KYSE-30, TE-10, and Eca-109) and human normal esophageal epithelial cells (HEEC). The results show that LINC00240 is strongly expressed in esophageal cancer cell lines, with the highest levels of expression in KYSE-30 and Eca-109 (Figure 7(b)). The above findings indicate that LINC00240 is remarkably expressed in esophageal cancer tissues and cell lines, implying that LINC00240 might play a vital regulatory part in the incidence and progression of esophageal cancer.

An interfering sequence targeting LINC00240 was constructed and then transfected into KYSE-30 and Eca-109 cells, and fluorescence qPCR was employed to identify the transfection efficiency. The outcome revealed in comparison to the blank control group (shRNA-NC), transfection of lentiviral vector knocking down LINC00240 could dramatically reduce the LINC00240 expression levels in esophageal cancer KYSE-30 and Eca-109 cells (Figures 7(c) and 7(d)).

### 3.8. Elevated LINC00240 Expression in the Plasma of Esophageal Cancer Patients

Fluorescence quantitative PCR was employed to determine LINC00240 expression levels in the preoperative plasma of esophageal cancer patients and a healthy control group. LINC00240 expression in plasma of esophageal cancer patients (3.94 ± 1.55) was found to be greater than that of normal controls (2.13 ± 0.89) (*P* < 0.01, Figure 8).

### 3.9. Correlation Analysis of LINC00240 Expression and Clinical Characteristics of Patients

Statistical analysis of clinicopathological data of 43 patients with esophageal cancer and expression of LINC00240 in plasma indicate that the expression level of LINC00240 was correlated with the degree of differentiation (*P*=0.0345) and TNM stage (*P*=0.0409) of patients as well as gender, age, and whether there is a vascular invasion or not. The results show no correlation between LINC00240 expression level and the location of the primary tumor or the number of the primary tumor (*P* > 0.05) (Table 1).

### 3.10. Knockdown of LINC00240 Can Considerably Inhibit the Progression of Esophageal Cancer Cells

The above-stated outcomes elucidated that LINC00240 expression was high in esophageal cancer cells. The highest-expression esophageal cancer cell lines KYSE-30 and Eca-109 were utilized to establish the knockdown LINC00240 model. The LINC00240 knockdown influence on the malignant ability of esophageal cancer cells KYSE-30 and Eca-10 was determined by the CCK-8 assay. The outcome demonstrated that LINC00240 knockdown considerably decreased the progression of esophageal cancer cells KYSE-30 and Eca-10 as to that of the blank control group (shRNA-NC) (Figure 9(a)). In addition, the outcomes of the plate clone formation assay reveal that LINC00240 knockdown markedly inhibited the clone formation property of esophageal cancer cells KYSE-30 and Eca-10 in comparison to the blank control group (shRNA-NC) (Figure 9(b)). The above outcome demonstrated that the LINC00240 knockdown could dramatically decrease the proliferation of esophageal cancer.

### 3.11. Knockdown of LINC00240 Can Significantly Inhibit Esophageal Cancer Cell Metastases

The above outcomes suggest that LINC00240 knockdown can greatly inhibit the progression of esophageal cancer cells. The Transwell assay was utilized to see if knocking out LINC00240 impacts the capability of esophageal cancer cells to metastasize. The number of cells migrating from the upper to lower chamber of Transwell on esophageal cancer cells KYSE-30 and Eca-10 reduced in the LINC00240 knockdown group as to that of the blank control group (shRNA-NC), indicating that the LINC00240 knockdown can considerably inhibit the migration ability of esophageal cancer cells (Figure 10). In order to further simulate the in vivo 3D environment, Matrigel gel was added to Tranwell. In comparison with the blank control group (shRNA-NC), the number of cells in LINC00240 knockdown esophageal cancer cells KYSE-30 and Eca-10 invading the lower chamber had decreased (Figure 10). The upper chamber results showed that LINC00240 knockdown could greatly decrease esophageal cancer metastases.

### 3.12. LINC00240 Regulates the Expression of miR-26a-5p through Competitive Binding in Esophageal Cancer Cells

The foregoing findings suggest that knocking off LINC00240 stops esophageal cancer cells from proliferating, invading, and migrating. For an in-depth study of the molecular mechanisms of LINC00240 regulating esophageal cancer cell activity, online bioinformatics prediction software was employed to predict the binding site of LINC00240. The binding site of LINC00240 and miR-26a-5p were found (Figure 11(a)). Esophageal cancer cells were transfected with synthetic miR-26a-5p mimics (mimics). The results of real-time quantitative PCR revealed that when compared to the blank control group (miR-NC), transfection of miR-26a-5p mimics (miR-26a-5p mimics) could significantly upregulate miR-26a-5p in esophageal cancer cells expression levels (Figure 11(b)). The miR-26a-5p expression in LINC00240 knockdown esophageal cancer cell lines was determined by real-time PCR. When compared to the blank control (shRNA-NC) group, the results demonstrated that knockdown of LINC00240 could significantly promote the miR-26a-5p expression level (Figure 11(c)). The luciferase gene activity assay further showed that in the LINC00240 wild-type group, compared with the miR-NC group, the addition of miR-26a-5p mimics could substantially inhibit the luciferase activity, while in the LINC00240 mutant group, the luciferase activity was significantly inhibited. Compared with the miR-NC group, the addition of miR-26a-5p mimics had no significant change in luciferase activity (Figure 11(d)). The expression level of LINC00240 in esophageal cancer (ESCA) tissue was strongly inversely linked with the expression level of miR-26a-5p (*r* = 0.002, *P* < 0.001), according to StarBase V3.0 data analysis (Figure 11(e)). The foregoing observations indicate that LINC00240 regulates miR-26a-5p expression in esophageal cancer cells via competitive binding.

### 3.13. Knockdown of LINC00240 Inhibits the Proliferation and Invasion of Esophageal Cancer by Negatively Regulating the Expression of miR-26a-5p

The above outcomes reveal that LINC00240 regulates the miR-26a-5p expression by competitive binding in esophageal cancer cells. To further investigate whether LINC00240 affects the malignant ability of esophageal cancer by modulating the miR-26a-5p expression, three experimental groups were set as follows: blank control group (shRNA-NC), knockdown LINC00240 group (shRNA-240), and knockdown LINC00240 (shRNA-240) + miR-26a-5p inhibitor group. The outcome of the plate clone formation assay showed that in comparison to the blank control group (shRNA-NC), knockdown of LINC00240 (shRNA-240) could dramatically decrease the number of plate clones formed in esophageal cancer cells. In contrast, knockdown of the LINC00240 (shRNA-240) + miR-26a-5p inhibitor group could significantly block the inhibitory effect of knockdown of LINC00240 (shRNA-240) on esophageal cancer cell plate clones (Figure 12(a)). Transwell experiments also demonstrated that in comparison to the blank control group (shRNA-NC), knockdown of LINC00240 (shRNA-240) could significantly inhibit the migration number of esophageal cancer cells. In contrast, LINC00240 (shRNA-240) + miR-26a-5p inhibitor group could significantly block the inhibitory effect of knockdown of LINC00240 (shRNA-240) on the migration ability of esophageal cancer cells (Figure 12(b)). The above results suggest that the knockdown of LINC00240 inhibits the proliferation and invasion of esophageal cancer by negatively regulating the expression of miR-26a-5p.

## 4. Discussion

Esophageal cancer pathology has been linked to a number of elements, according to research. Long noncoding RNAs (lncRNAs) are suspected of having an essential part in the evolution of various forms of cancers in recent years, thanks to the advent of high-throughput gene sequencing technologies [15, 16]. lncRNAs have been involved in regulating physiological functions such as cell proliferation, differentiation, metastasis, and apoptosis, along with the incidence and development of numerous malignant tumors, according to previous research [7, 9]. For example, lncRNACASC9 encourages the metastases of ESCC (esophageal squamous cell carcinoma) by interacting with CREB-binding protein to upregulate LAMC2 expression [17]. Also, lncRNAs in peripheral blood can be used as efficient, noninvasive biological indicators for diagnosing esophageal cancer [18]. Therefore, identifying and studying new lncRNAs is extremely important for diagnosing cancer in its early stages, monitoring postoperatively, and treating esophageal cancer.

As sequencing and omics technologies have advanced, there have been more opportunities to investigate potential diagnostic and therapeutic targets and gain a deeper understanding of the mechanism underlying esophageal cancer. In the present research, we combined bioinformatics analysis and in vitro experiments to explore the role of LINC00240 in the occurrence and progression of esophageal cancer and the possible mechanism. In the TCGA database, we found that LINC00240 is elevated in esophageal cancer. To individually predict the 1-, 3-, and 5-year survival probabilities of patients with esophageal cancer, we constructed a predictive model based on the results of multivariate analysis in the database. The result prediction model has a certain accuracy. Further data analysis in the TIMER database supports that the LINC00240 expression may be considerably related to tumor immune infiltration and indicates that LINC00240 might have a significant function in promoting immune escape of tumor cells in the esophageal cancer tumor microenvironment. Next, we analyzed the correlation between LINC00240 and the target molecules related to current esophageal cancer targeted drug therapy. We found that LINC00240 has a good correlation with EGFR, VEGFA, VEGFB, VEGFC, VEGFD, ERBB2, and MSI1. The results can provide a better reference for the selection of targeted drugs from the side. There are also relevant reports in relevant global clinical trials. For example, AdvanTIG-203 shows that tislelizumab combined with TIGIT monoclonal antibody Ociperlimab has better advantages compared with placebo in the treatment of PD-L1 positive esophageal squamous cell carcinoma. The Keynote-590 study showed that in Chinese patients with advanced esophageal cancer, pembrolizumab combined with chemotherapy can significantly improve patient survival, progression-free survival, and objective response rate compared with chemotherapy. RATIONALE 302 study showed that compared with second-line chemotherapy, tislelizumab can significantly improve the survival time of patients with advanced or metastatic esophageal squamous cell carcinoma whose disease has progressed after first-line therapy and has a higher response rate, longer response time, and lower adverse reactions. RAMONA study also proposes that nivolumab combined with ipilimumab is safe and feasible in the second-line treatment of elderly patients with esophageal squamous cell carcinoma. Therefore, immunotherapy combined with targeted therapy may be a better treatment option for recurrent or metastatic esophageal cancer. Moreover, the molecule LINC00240 studied in this project is not only related to the immune infiltration of esophageal cancer but also to the target molecule, which reflects that our research has certain clinical value.

Then, through GSEA enrichment analysis, it was observed that LINC00240 may influence the biological events of esophageal cancer through five pathways: KEGG_APOPTOSIS; KEGG_VEGF_SIGNALING_PATHWAY; WP_ EGFEGFR_SIGNALING_PATHWAY; REACTOME_ CELL_CYCLE_CHECKPOINTS. Previous studies also showed that LINC00240 promoted the proliferation, migration, and EMT of gastric cancer cells through the miR-124-3p/DNMT3B axis; lncRNA LINC00240 inhibited the invasion and migration of non-small-cell lung cancer by sponging miR-7-5p. Therefore, cytological experiments further verified the expression of LINC00240 in esophageal cancer.

This research observed that LINC00240 is largely present in esophageal cancer cells, and knocking down LINC00240 can strongly ameliorate the cancer cell growth, clone formation, and malignant abilities of esophageal cancer cells. According to molecular mechanism studies, endogenous LINC00240 inhibits the buildup and invasion of esophageal cancer cells by combining and modulating the miR-26a-5p expression.

The uncontrolled, unlimited proliferation ability of cancerous cells is the main element in causing poor prognosis for patients. Searching for drugs, oncogenes, lncRNAs, or other targets that block the rapid division of cancerous cells is one of the hotspots in tumor research. For example, stable knockdown of DLL4 decreases the esophageal cancer metastases by attenuating Akt phosphorylation [19]. lncRNA SNHG7 expression is considerably increased in esophageal cancer cells, and it can promote esophageal cancer growth by influencing the expression of p15 and p16 [20]. LINC00240 is a recent discovery of a novel family of lncRNAs that regulates the onset and progression of various cancers. LINC00240, for example, is elevated in gastric cancer cells, and its increased levels are linked to a higher TNM stage, more distant and metastatic lymph nodes, with awful health and low chances of illness-free survival [21]. lncRNA LINC00240 represses malignant abilities of non-small cell lung cancer by controlling miR-7-5p [22]. Through the miR-124-3p/DNMT3B axis, LINC00240 can also enhance the metastases of gastric cancer [12]. LINC00240 was discovered to be substantially present in esophageal cancer tissues in the present research. Further in vitro cell function investigations revealed that knocking down LINC00240 greatly inhibited the rapid growth of esophageal cancer cells and the number of plate clones, suggesting that LINC00240 in esophageal cancer may be a cancer-promoting agent gene, providing new targets for subsequent targeted therapy. Inhibiting the expression of LINC00240 can greatly suppress the metastases of esophageal malignant cells.

Previous research studies have revealed that miR-26a-5p exhibits various modulatory functions in different tumor tissues, acting as an antitumor, or tumor promoter. For example, as a tumor suppressor gene, miR-26a-5p has lower levels in gastric cancer tissue. Overexpression of miR-26a-5p can suppress the Wnt5a expression, thereby promoting programmed cell death and inhibiting the malignant capabilities of gastric cancer cells [23]. On the other hand, among the prooncogenes, miR-26a-5p acts as an oncogenic microRNA in non-small-cell lung cancer by targeting FAF1 and might function as a possible therapeutic target [24]. Analysis of miR-26a-5p expression levels in plasma helps to differentiate bladder cancer patients from healthy controls [25]. The findings of this research further demonstrate that LINC00240 can negatively regulate the miR-26a-5p expression in esophageal cancer cells. Cell function experiments demonstrated that inhibiting miR-26 knocked down the expression of LINC00240. However, the further molecular mechanism, that is, how miR-26a-5p controls downstream target gene expression to exert its tumor suppressor effect, needs to be further studied and verified by in vivo experiments.

## Figures and Tables

**Figure 1:** Elevated expression of LINC00240 in esophageal cancer. (a) LINC00240 expression in pan-cancer. (b) Expression of LINC00240 in unpaired tissues of esophageal cancer (tumor 162 cases—normal 11 cases). (c) ROC analysis of LINC00240 showed some discrimination ability among the tumor and normal tissue. Note: ^*∗*^*P* < 0.05; ^*∗∗*^*P* < 0.01; ^*∗∗∗*^*P* < 0.001.

**Figure 2:** Nomogram and calibration plot. (a) Nomogram used to predict 1-, 30, and 5-year OS probability in patients suffering from esophageal cancer.

**Figure 3:** (a) LINC00240 was considerably linked to immune cell infiltration in the TIMER database. (b) LINC00240 expression was considerably associated with immune cell infiltration in esophageal cancer. ^*∗*^*P* < 0.05; ^*∗∗*^*P* < 0.01; ^*∗∗∗*^*P* < 0.001.

**Figure 4:** Correlation between LINC00240 and molecular targeted therapy drug target molecules in the TCGA database.

**Figure 5:** Coexpressed gene analysis of LINC00240. (a) Heatmap illustrating the top 50 genes positively correlated with LINC00240 in esophageal cancer; (b) heatmap depicting the top 50 genes negatively correlated with LINC00240 in esophageal cancer.

**Figure 6:** Six related pathways that LINC00240 may be involved in esophageal cancer. The gene ear biology biological process gene set from MSigDB was employed. 1500 random sample permutations were performed. NES: normalized enrichment score; NOM-p: nominal *P*-value; FDR-q: false discovery rate.

**Figure 7:** LINC00240 is highly expressed in cell lines. (a) Fluorescence quantitative PCR detects LINC00240 expression in 45 esophageal malignant tissues and paracancours tissues. (b) Fluorescence quantitative PCR detects LINC00240 in esophageal cancer cell lines. (c, d) Fluorescence quantitative PCR detection of transfection effect after knockdown of LINC00240 in esophageal cancer cell lines (KYSE-30 and Eca-109); ^*∗∗*^*P* < 0.01.

**Figure 8:** The expression level of LINC00240 in preoperative plasma of patients with esophageal cancer detected by real-time PCR, ^*∗∗*^*P* < 0.01.

**Figure 9:** LINC00240 Knockdown blocks the progression of esophageal cancer cells. (a) CCK-8 assay detected the LINC00240 knockdown effect on the rapid growth of esophageal cancer cells. Effect of ability, ^*∗∗*^*P* < 0.01.

**Figure 10:** Knockdown of LINC00240 inhibits the invasion and migration (100×) of esophageal cancer cells; ^*∗*^*P* < 0.05; ^*∗∗*^*P* < 0.01.

**Figure 11:** LINC00240 regulates the miR-26a-5p expression by competitive binding in esophageal cancer cells. (a) Online bioinformatics software predicts that LINC00240 has a binding site with miR-26a-5p, (b) real-time quantitative PCR detection in transfection efficiency of miR-26a-5p mimics in esophageal cancer cells, (c) real-time quantitative PCR detection of the effect of knockdown of LINC00240 on the miR-26a-5p expression in esophageal cancer cells, (d) detection of luciferase activity and the binding activity of INC00240 to miR-26a-5p in esophageal cancer cells, and (e) StarBase V3.0 data analysis of the relation between the LINC00240 expression and the miR-26a-5p expression in esophageal cancer (ESCA) tissue, ^*∗∗*^*P* < 0.01.

**Figure 12:** Knockdown of LINC00240 inhibits plate clone formation (a) and invasive ability (100×) (b) of esophageal cancer by negatively regulating the expression of miR-26a-5p; ^*∗*^*P* < 0.05; ^*∗∗*^*P* < 0.01.

**Table 1:** Expression and clinical features of esophageal cancer patients analyzed for correlation.

Characteristics	*N*	LINC00240 expression	*P*
Gender			
Male	26	3.81 ± 1.73	0.6224
Female	17	4.16 ± 2.89	
Age			
<60	9	3.51 ± 1.34	0.4569
≥60	34	3.98 ± 1.74	
Invasion into lymph			
Yes	33	4.11 ± 1.28	0.1985
No	10	3.53 ± 1.03	
Diameter of tumor (cm)			
<5	12	3.49 ± 1.12	0.1196
≥5	31	4.23 ± 1.45	
Differentiated degree			
Well-differentiated	15	3.51 ± 1.34	**0.0345**
Low differentiation	28	4.63 ± 1.72	
TNM stage			
*T*1 + *T*2	34	3.04 ± 1.63	**0.0409**
*T*3 + *T*4	9	4.39 ± 1.99	
Vascular invasion			
Yes	11	3.98 ± 1.23	0.1719
No	32	3.44 ± 1.07	
Number of primary lesions			
Single	27	3.89 ± 1.17	0.4792
Multiple	16	4.17 ± 1.36	

## Data Availability

The data are available from the corresponding author upon request via e-mail (chengchun2002@ntu.edu.cn).
